# Region Matching of SAR Images Using Blocks for Target Recognition

**DOI:** 10.1155/2021/5410440

**Published:** 2021-09-29

**Authors:** Chao Shan, Minggao Li, Zihao Chen, Lei Han

**Affiliations:** Department of Special Operations Medicine, The Sixth Medical Center of Chinese PLA General Hospital, Beijing 100048, China

## Abstract

A synthetic aperture radar (SAR) target recognition method based on image blocking and matching is proposed. The test SAR image is first separated into four blocks, which are analyzed and matched separately. For each block, the monogenic signal is employed to describe its time-frequency distribution and local details with a feature vector. The sparse representation-based classification (SRC) is used to classify the four monogenic feature vectors and produce the reconstruction error vectors. Afterwards, a random weight matrix with a rich set of weight vectors is used to linearly fuse the feature vectors and all the results are analyzed in a statistical way. Finally, a decision value is designed based on the statistical analysis to determine the target label. The proposed method is tested on the moving and stationary target acquisition and recognition (MSTAR) dataset and the results confirm the validity of the proposed method.

## 1. Introduction

High-resolution synthetic aperture radar (SAR) images provide basis for efficient and accurate intelligence interpretation [1]. The moving and stationary target acquisition and recognition (MSTAR) dataset provided a benchmark for the research and evaluation of SAR target recognition algorithms [2, 3]. The resolution of SAR images in this dataset reaches 0.3 m, which can be effectively used for the classification of vehicle targets such as tanks, armored vehicles, and cannons. With nearly 30 years of developments, the SAR target recognition methods on the MSTAR dataset have made great progress in performance. However, these researches also revealed the shortcomings of current methods for the extended operating conditions (EOCs). EOCs in SAR target recognition may be caused by variations of target configurations, backgrounds, sensors, etc. [4]. As a result, the test samples to be recognized may have notable differences with the established training samples. Hence, the recognition problems under the standard operating condition (SOC) are not challenging and more focus should be imposed on solving the nuisance cases under EOCs [5, 6].

SAR target recognition methods usually combine feature extraction and classifier design. The two steps are closely coupled to improve the recognition performance. In terms of feature extraction, a rich set of features has been applied into SAR target recognition, which can be generally summarized as geometrical, transformation, and electromagnetic ones. The geometrical features depict target shapes including region, contour, and shadow. In [7–10], the Zernike and Chebyshev moments were used as basic features to describe the target region. In [11–13], the target regions in SAR images are directly matched with the support of morphological operations. In [14–16], the target contour or outline was adopted for target recognition. The transformation features are usually extracted based on the pixel distribution in SAR images. Typical algorithms include the projection ones such as principal component analysis (PCA) [17] and nonnegative matrix factorization (NMF) [18] and the decomposition ones such as monogenic signal [19, 20] and empirical mode decomposition (EMD) [21]. The electromagnetic features describe the backscattering characteristics of the targets such as the attributed scattering centers (ASC) and polarization [22–25]. In the classification stage, a decision is made on the features extracted from the test sample. For the transformation features with uniform forms and dimensions, traditional classifiers such as K-nearest neighbor (KNN) [17], support vector machine [26, 27] (SVM), and sparse representation classification (SRC) [27–29] can be directly employed for classification. For the irregularly arranged and inconsistent features such as target contour points and scattering centers, it is necessary to employ some specially designed classification strategies, such as the similarity measure for the scattering center sets designed in [22–25]. In recent years, the deep learning models have been also widely used in SAR target recognition like the convolutional neural networks (CNN) [30–32]. The deep learning models are directly trained and learned based on the original images, avoiding the traditional manual feature extraction process. The research results verified the effectiveness of the deep learning models for SAR target recognition under the premise of sufficient training samples. For EOCs, the relevant training samples are very limited, which leads to poor adaptability of the deep learning methods for SAR target recognition.

This paper proposes a SAR target recognition method based on image blocking and matching. The original image is separated into several blocks and the target label is determined by comparing and analyzing each block. Under EOCs, the target in SAR images may have local changes caused by noises, occlusions, etc. But in essence, the corrupted test sample can still share high similarities with the corresponding sample from the actual training class. In this sense, by observing and evaluating the local differences and consistency between SAR images, EOCs can be overcome with high effectiveness. The proposed method divides the SAR image into 4 blocks of equal area with the target center as the reference point. For each block, the monogenic signal is employed for feature extraction and a unified feature vector is constructed. According to the properties of monogenic signal, the constructed features can effectively reflect the spectral characteristics and local distribution of the target. For the feature vector constructed from each block, SRC is used for as the basic classifier and the reconstruction error vector of different training classes can be obtained. For the results of 4 blocks, a random weight matrix with massive weight vectors is developed to linearly fuse them. For the correct class, the blocks with low reconstruction errors account for the majority, so its corresponding reconstruction errors from the four blocks have smaller mean and variance. On the contrary, for the wrong class, the mean value of the four reconstruction errors tends to be relatively large and also the variance because of the randomness. Based on statistical analysis, a decision value is defined as the measure to determine the target label. In the experiments, the proposed method is investigated on the MSTAR dataset under different scenarios. The experimental results show its significant superiority over the compared methods under both SOC and EOCs.

## 2. SAR Image Blocking

The previous researches showed that EOCs in SAR images are mostly related to the local variations of the target. For example, in the case of configuration variation, the test target only has some local structural differences with the reference one in the training set, which can also be reflected in local pixel distribution and geometric structure in the SAR image. Therefore, it is meaningful to fully investigate the local changes of the target as for handling the EOCs. Traditional methods were generally developed based on overall SAR images for feature extraction and classification. In this case, the local changes may cause variations of global feature changes. As a result, the idea of global feature matching may lose some precision for target classification. As a remedy, this study divides the original SAR image into several blocks and then analyzes the target characteristics by each of them separately. Finally, a reliable classification result can be achieved based on the joint analysis of the results from different blocks.

Specifically, the image blocking algorithm used can be implemented mainly in two steps. First, the original image is centralized and the target centroid is adopted as the reference point for the following blocks. Afterwards, the original image is divided along the range and cross range directions to obtain 4 subimages.  Figure 1 shows the blocking result of a SAR image from the MSTAR dataset. Each subimage is processed independently. Hence, when a certain subimage has some local variations, its classification result has little influence on other subimages. It is beneficial to obtain the true correlation between the test sample and the training classes, thus improving the classification accuracy.

## 3. Feature Extraction

For each subimage from the blocking stage, the traditional target recognition procedure with feature extraction and classification is employed. The monogenic signal is used for feature extraction for those subimages [19, 20]. Denote *z*=(*x*, *y*)^T^ as the coordinates in 2D space; *f*(*z*) is the image or matrix to be processed. The monogenic signal corresponding to *f*(*z*) is calculated as follows:

(1) $$\begin{array}{c} f_{M}\left(z\right)=f\left(z\right)-\left(i,j\right)f_{R}\left(z\right), \end{array}$$

where *f*_*R*_(*z*) represents the Riesz transform of *f*(*z*); *i* and *j* are the imagery units along two dimensions of the image. A further decomposition is conducted with three types of components, i.e., local amplitude, local phase, and local orientation, as follows:

(2) $$\begin{array}{c} \text{amplitude}:A\left(z\right)=\sqrt{f{\left(z\right)}^{2}+{\left|f_{R}\left(z\right)\right|}^{2}},\\ \text{phase}:\varphi \left(z\right)=a\;\tan\;2\left(\left|f_{R}\left(z\right)\right|,f\left(z\right)\right)\in \left(-\pi ,\pi \right],\\ \text{orientation}:\theta \left(z\right)=a\;\tan\;2\left(\frac{f_{y}\left(z\right)}{f_{x}\left(z\right)}\right)\in \left(-\frac{\pi }{2},\frac{\pi }{2}\right], \end{array}$$

where *f*_*x*_(*z*) and *f*_*y*_(*z*) are resulted from the *i*-imaginary and *j*-imaginary parts of *f*_*M*_(*z*), respectively.

Generally, the target recognition methods based on monogenic signal are developed on the three components because they can comprehensively describe the target chrematistics. *A*(*z*) reflects the local amplitudes, which describes the intensity distribution. *φ*(*z*) and *θ*(*z*) depict the structural and geometric properties of the target, respectively. This study constructs a feature vector based on the monogenic components with reference to [15], in which the special parameters were determined for monogenic decomposition and the results are reorganized to a concatenated vector.

## 4. Method Description

### 4.1. SRC

For the extracted monogenic features, SRC is adopted as the classifier [27–29]. The idea of sparse representation assumes that the test sample can be linearly reconstructed by the training samples from the same class. Φ_*k*_=[*x*_*k*,1_,…, *x*_*k*,*n*_*k*__] ∈ *R*^*d*×*n*_*k*_^(*k*=1,…, *C*) is constructed as a local dictionary with *n*_*k*_*d*-dimensional samples from the *k*th class; the test sample *y* is represented as follows:

(3) $$\begin{array}{c} y=x_{k,1}\alpha_{k,1}+\cdots +x_{k,n_{k}}\alpha_{k,n_{k}}=\Phi_{k}\alpha_{k}, \end{array}$$

where *α*_*k*_=[*α*_*k*,1_,…,*α*_*k*,*n*_*k*__]^*T*^ ∈ *R*^*n*_*k*_^ comprises of the linear coefficients.

When the test sample is from an unknown class, the linear representation should be performed on all the potential classes. So, SRC usually conducts the representation over the global dictionary as follows:

(4) $$\begin{array}{c} \hat{\alpha }=\underset{\alpha }{\arg\min}{\left\|\alpha \right\|}_{0},\\ \text{s.t. }{\left\|y-\Phi \alpha \right\|}_{2}^{2}\leq \varepsilon , \end{array}$$

where Φ=[Φ_1_,…, Φ_*C*_] ∈ *R*^*d*×*n*^ is the global dictionary which comprises of samples from *C* training classes; *α*=[*α*_1_,…,*α*_*C*_]^*T*^ ∈ *R*^*n*^ is the global coefficient vector to be solved; *ε* is the error tolerance.

As a nondeterministic polynomial (NP) hard problem, the optimization task in equation (4) is complex to be solved. There are two main ways to handle this issue in previous works. One is replacing the *ℓ*_0_ norm by *ℓ*_1_ norm to formulate a convex optimization objective function for smooth solution. Another is using the greedy algorithms, such as the orthogonal matching pursuit (OMP), to obtain an approaching result.

### 4.2. Decision Fusion with Random Weight Matrix

For the classification results from different subimages, they should be combined and fused to reach a final decision. Although there are different information fusion algorithms in previous works, the linear weighing fusion is a simple but suitable one for this study. Furthermore, to handle the possible instability of a fixed weight vector, the random weight matrix *W* is designed with multiple choices of weight vectors, in which the elements in each row are subject to the following constraint:

(5) $$\begin{array}{c} w_{0}+w_{1}+\cdots +w_{n}=1. \end{array}$$

For different weight vectors in the weight matrix, disproportionate importance is imposed on different subimages. With a rich set of weight vectors, the complex situations in different subimages can be comprehensively analyzed. The fusion process with the random weight matrix is performed as follows:

(6) $$\begin{array}{c} FV_{k}=W*RV_{k}. \end{array}$$

Here, *RV*_*k*_ denotes a row vector related with the *k*th training class, containing *N* elements corresponding to reconstruction errors of the *N* subimages. *FV*_*k*_ corresponds to the fused error vector at different choices of random weight vectors. Then, for *C* different training classes, there are *C* fused vectors denoted as *FV*_1_, *FV*_2_,…, *FV*_*C*_.

When the test sample is actually from the *k*th class, the fused errors in *FV*_*k*_ tend to be small. Otherwise, these errors are probably at high levels. In addition, the errors at different weight vectors may vary intensively and disorderly. These statistical phenomena can be used to evaluate the true relationship between the test sample and training classes. At first, the mean and variance of *FV*_*k*_ are calculated as *μ*_*k*_=mean(*FV*_*k*_) and *σ*_*k*_^2^=Var(*FV*_*k*_). Then, a similarity measure is developed as follows to properly evaluate the relation between the test sample and *k*th training class:

(7) $$\begin{array}{c} S_{k}=\frac{1}{\mu_{k}}*\;\exp\left(\frac{\sigma_{k}^{2}}{2}\right). \end{array}$$

Accordingly, with lower *μ*_*k*_ and *σ*_*k*_^2^, a higher *S*_*k*_ can be achieved, which indicates a higher similarity. After obtaining the similarities between the test sample and different classes, the target label can be determined as follows:

(8) $$\begin{array}{c} \text{indentity}\left(Y\right)=\underset{k}{\max}\left(S_{k}\right),\;k=1,2,\ldots ,C. \end{array}$$

Figure 2 shows the basic implementation process of the proposed method. The image blocking algorithm is used to process all training samples, and a single feature vector is extracted for each subimage based on the monogenic signal. Afterwards, the dictionaries of different subimages are constructed. For the test sample, the same blocking algorithm is used for processing and feature extraction. Then, the corresponding four monogenic feature vectors are obtained. SRC is used to classify the feature vectors of the 4 blocks, and the reconstruction error vectors are obtained. Finally, the 4 error vectors are fused using the random weight matrix and the target label of the test sample is determined.

## 5. Experiments and Analysis

### 5.1. Basics of MSTAR Dataset

The experiments are designed and conducted based on the MSTAR dataset, a popular and authoritative data source for the evaluation of SAR target recognition algorithms. Ten typical targets shown as Figure 3 are measured with thousands of 0.3 m-resolution SAR images, which is suitable to be used for target identification. With the support of the rich set of SAR images, various conditions or situations can be designed for experimental validations.

To objectively evaluate the performance of the proposed, we also drawn several previous methods in this field for comparison. The first one used Zernike moments of the whole target as features, which were classified by SVM for decision [7]. The second one adopted the monogenic signal and the resulted three types of features were classified by joint sparse representation [20]. The third one employed the ASCs as features and developed a matching algorithm [23]. The fourth one developed a novel CNN architecture, namely, all fully convolutional neural network (A-ConvNet), for SAR target recognition [31], which is chosen as a representation for deep learning-based algorithms. The following tests are conveyed under both SOC and EOCs to provide comprehensive evaluation of the proposed method.

### 5.2. Condition 1: SOC

As explained in the former texts, SOC is a simple but representative case in SAR target recognition.  Table 1 establishes the setup for SOC based on the MSTAR dataset. The training and test samples with 2° depression angle variance are assumed to be highly alike.  Figure 4 displays the recognition results of the proposed method with a confusion matrix. As shown, the *x* and *y* labels correspond to the 10 targets and the diagonal elements mark the recognition rates of different classes. We define the average recognition rate of the 10 classes as *P*_av_=(*N*_C_/*N*_*T*_), in which *N*_C_ denotes the number of the correctly-classified samples and *N*_T_ is the total number of all test samples. Correspondingly, the *P*_av_ of the proposed method is computed as 99.48%.  Table 2 summarizes the *P*_av_*s* of all the methods. In comparison with the Zernike method, the blocking of the whole image and decision fusion significantly enhance the final result. Compared with the monogenic method, the joint use of the blocks further improves the recognition performance. The A-ConvNet method ranks second in these methods, validating the high effectiveness of deep learning models when the test samples share high similarities with the training ones.

### 5.3. Condition 2: Configuration Variants

For the ground targets, it is usual to see their variants for different scenarios. The 10 targets in the MSTAR dataset also have configuration variants and some are chosen as shown in Table 3 to establish the experimental setup. For the BMP2 and T72 targets, their test samples include more configurations than the training sets. The use of BTR70 in this case is mainly causing confusion, thus enhancing the difficulty of the recognition problem.  Table 4 lists the *P*_av_*s* of different methods for comparison. With the highest performance, the proposed method maintains the best robustness under configuration variants. The ASC matching method ranks second among the five methods. As local descriptors, the structural modifications caused by configuration variants can be well sensed by the ASC parameters. Compared with the Zernike and monogenic methods, the blocking and fusion strategy in the proposed method contributes to higher recognition performance.

### 5.4. Condition 3: Depression Angle Variances

When the test samples and the training samples come from two depression angles with large differences, their similarity also decreases sharply, enhancing the difficulty of the recognition problem.  Table 5 establishes the experimental setup for configuration variants. The training samples of the three targets are from 17° depression angle, but the corresponding test samples are from 30° and 45°, respectively.  Figure 5 shows the performance of all the methods at the two depression angles for comparison. First, the performance at 30° depression angle is much higher than that at 45°, which shows that the large depression angle change causes intensive influences on the recognition results. Second, at both depression angles, the proposed method achieves the highest *P*_av_*s* because the blocking patches could better deal with the image variations caused by depression angle changes. In the reference methods, the ASC matching method obtains the best performance due to the robustness of features.

### 5.5. Condition 4: Noise Corruption

When the test sample is measured with a low signal-to-noise ratio (SNR), it is assumed to have many differences with the one from a high SNR. The original MSTAR images were mainly acquired from high SNRs. To test the method under noise corruption, we first simulate the noisy test sets based on the original test samples. The energy of the original SAR image is used as the reference and the additive Gaussian noises are generated according to the desired SNR [24]. Finally, these noises are added into the SAR images to obtain the noisy image. Based on the noisy test sets at different SNRs, the performance of all the methods is obtained, as shown in Figure 6. It is noticeable that the noises have significant influences on the recognition performance of all the methods. In comparison, the proposed method achieves the highest *P*_av_*s* at different noise levels, validating its superior noise robustness. The blocking algorithm divides the whole image into several patches. The noises in one parch will not affect the other ones. Therefore, the noise interferences can be relieved to some extent. In addition, the monogenic features have some robustness to noises. So, the overall noise robustness of the proposed method can be further enhanced.

### 5.6. Condition 5: Partial Occlusion

The possible occlusion case is also considered in the experiments. For example, when there is a building or obstacles between the target and SAR sensor along the radar view direction, some parts of the target may be occluded and will not be reflected in the measured SAR image. According to the previous works, the directional occlusion model is adopted in this experiment [24]. A certain proportion of the target region is removed from the original image to generate the occluded sample. Based on the simulated test sets at different occlusion levels, the performance of all the methods is obtained, as shown in Figure 7. Similar to the case of noise corruption, the directional occlusions decrease the recognition performance. With the highest *P*_av_*s* at different occlusion levels, the good robustness of the proposed method is validated. With the blocked patches, the occlusions in one of them will not affect the remaining ones. In this sense, the occlusions can be better handled to make sure the fused decision is more accurate.

## 6. Conclusion

The paper proposes a SAR image target recognition method based on block matching. The original SAR image is processed in 4 blocks, and each subblock reflects local characteristics in different directions. The monophonic signal is used to describe the spectral characteristics and local features of each subblock and construct a feature vector. The monomorphic feature vectors of the 4 subblocks are classified by SRC to obtain the reconstruction error vector. Based on the random weight matrix, the reconstruction error vectors of the 4 subblocks are weighted and fused. Through statistical analysis of the fusion results under multiple sets of weight vectors, the decision variables are designed to obtain sample categories. The experiment sets 4 test conditions in the MSTAR dataset, including standard operating conditions and extended operating conditions. The experimental results show that this method has significant performance advantages compared with the existing methods.

## Figures and Tables

**Figure 1:** Illustration of the results of blocking a SAR image.

**Figure 2:** Procedure of implementation of the proposed method.

**Figure 3:** The ten targets in MSTAR dataset. (a) BMP2. (b) BTR70. (c) T72. (d) T62. (e) BRDM2. (f) BTR60. (g) ZSU23/4. (h) D7. (i) ZIL131. (j) 2S1.

**Figure 4:** Confusion matrix of the proposed method under SOC.

**Figure 5:** Comparison between the performance of the proposed method and reference ones under depression angle variances.

**Figure 6:** Comparison between the performance of the proposed method and reference ones under noise corruption.

**Figure 7:** Comparison between the performance of the proposed method and reference ones under partial occlusion.

**Table 1:** Details of training and test samples under SOC.

Type	Training set		Test set	
	Depression angle (°)	Number of samples	Depression angle (°)	Number of samples
BMP2	17	233	15	195
BTR70		233		196
T72		232		196
T62		299		273
BRDM2		298		274
BTR60		256		195
ZSU23/4		299		274
D7		299		274
ZIL131		299		274
2S1		299		274

**Table 2:** Comparison between the performance of the proposed method and reference ones under SOC.

Method	Proposed	Zernike	Monogenic	ASC	A-ConvNet
*P*_av_ (%)	99.48	98.12	98.86	98.54	99.14

**Table 3:** Details of training and test samples under configuration variants.

Type	Training set			Test set		
	Depression angle (°)	Configuration	Number of samples	Depression angle (°)	Configuration	Number of samples
BMP2	17	9563	233	15	9566	196
					c21	196

BTR70	17	c71	233	15	c71	196

T72	17	132	232	15	812	195
					s7	191

**Table 4:** Comparison between the performance of the proposed method and reference ones under configuration variants.

Method	Proposed	Zernike	Monogenic	ASC	A-ConvNet
*P*_av_ (%)	98.64	97.92	97.61	98.02	97.83

**Table 5:** Details of training and test samples under depression angle variances.

Type	Training set		Test set	
	Depression angle (°)	Number of samples	Depression angle (°)	Number of samples
2S1	17	299	30	288
			45	303
BRDM2		298	30	287
			45	303
ZSU23/4		299	30	288
			45	303

## Data Availability

The dataset can be accessed upon request to the corresponding author.
